# Does Development Assistance for Health Really Displace Government Health Spending? Reassessing the Evidence

**DOI:** 10.1371/journal.pmed.1001214

**Published:** 2012-05-08

**Authors:** Rajaie Batniji, Eran Bendavid

**Affiliations:** Stanford University, Stanford, California, United States of America

## Abstract

Rajaie Batniji and Eran Bendavid dispute recent suggestions that health aid to developing countries leads to a displacement of government spending and instead argue that current evidence about aid displacement cannot be used to guide policy.

**Summary Points**

- At the core of the current aid debate is the question of whether development assistance for health provided to developing country governments increases health expenditures.
- It has recently been suggested that development assistance for health to governments leads to a displacement of government spending, reinforcing skepticism about health aid.
- Here we examine a database of public financing for health from 1995 to 2006 and demonstrate that prior conclusions drawn from these data are unstable and driven by outliers.
- While government spending may be displaced by development assistance for health in some settings, the evidence is not robust and is highly variable across countries. We recommend that current evidence about aid displacement cannot be used to guide policy.

## Re-thinking Aid Displacement in the Health Sector

There has been considerable concern in the international development community about aid displacement in the health sector. That is, a concern that foreign aid to the health sector leads to a displacement or diversion of government funds from the health sector. Foreign aid, also known as development assistance, includes funding from international development agencies in donor countries, multilateral agencies like the World Bank and Global Fund, and private sources. The concern about displacement penetrates questions about the strings attached to aid, the monitoring of aid, and whether aid should be given to governments in the first place. A core question being asked is, does development assistance for health increase health spending? Or, do aid funds merely displace government funding for health?

## Questioning the Argument That Health Aid Leads to Reduced Government Investment in Health

Concerns about aid displacement are as old as development assistance. As a leading World Bank economist famously said in 1947, “When the World Bank thinks it is financing an electric power station, it is really financing a brothel.” [1] More recently, experts commenting in the press have suggested, “When an aid official thinks he [sic] is helping a low-income African patient avoid charges at a health clinic, in reality, he is paying for a shopping trip to Paris for a government minister and his wife [2].” The concerns—and the cynicism— about foreign aid being displaced and diverted for less-than-noble purposes have been in place the last 60 years.

Some analysis has been done to assess the scale of aid displacement in different sectors and countries. In one analysis, World Bank economists examined aid to 18 African countries from 1971 to 1995, and found that for every US dollar of aid received, government spending increased by US$0.90 [1]. That study also found that some aid intended for capital improvements, like the building of hospitals, went to operations and to the repayment of past loans. But across sectors and regions, the evidence for aid displacement is mixed. For example education aid was found to have no discernible effect on education spending worldwide; however, each US dollar in education aid in Africa led to nearly US$1.00 increase in education spending [1].

Country analyses have also identified great variation in the extent of displacement. One study showed that aid to India “merely substitutes for spending that the government would have undertaken anyway,” concluding that “funds freed by aid are spent on non-development activities [3].” In contrast, a study of aid to Vietnam's transportation sector found that aid stayed within that sector [4].

Recently, attention has turned to whether health aid increases government health spending. In 2009, Farag and colleagues found that from 1995 to 2006, each US dollar increase in development assistance for health (DAH) to low-income countries was associated with a US$0.14 decrease in government health spending [5]. A subsequent analysis by Lu and colleagues made the case that for every additional US dollar of DAH from 1995 to 2006, government health expenditures from domestic sources fell by at least US$0.43 [6]. This latter study is referenced frequently in conversations with decision-makers at aid agencies as a cautionary note about DAH. The analysis appears to have reinforced skepticism about health aid.

A closer look at the analysis by Lu and colleagues, using data made available in May 2011 [7], shows that the association between DAH and displacement of government health expenditures is not robust after exclusion of a small subset of data. The trends are driven by outliers, and country data cluster and follow widely divergent trends (Figure 1). The primary finding by Lu and colleagues, which we are challenging here, is the negative relationship between government health expenditure (GHE-S)/gross domestic product (GDP) and DAH-Gov/GDP. GHE-S/GDP is government health spending from domestic sources as a percentage of GDP for a country in each year from 1995 to 2006. DAH-gov/GDP is development assistance for health disbursed to government as a percentage of GDP for each country in each year from 1995 to 2006. Using Lu and colleagues' data on government health spending and Institute for Health Metrics and Evaluation (IHME) data on DAH [8], we replicated their results and found that the linear relationship between DAH and government health expenditure from domestic sources is lost when country-years in which World Health Organization (WHO) and International Monetary Fund (IMF) estimates differ by 10-fold or more are removed, when a small set of implausible data points are removed, and when restricting the sample to eliminate those countries that receive very little DAH as a percentage of GDP. In sum, any linear relationship that exists among the data is too tenuous to be a basis for policy.

**Figure 1:** Primary data scatter of the relationship between DAH and GHE-S in all countries. Both DAH and GHE-S are presented here as a percentage of GDP, with GHE-S based on IMF data. Each point on the above plot represents a country-year observation used in the analysis. Data source: IHME [2].

## Re-evaluating the Data: Inconsistencies and Omissions

Much debate surrounded the initial publication of the paper by Lu and colleagues, but those engaged in the correspondence acknowledged that they were challenging neither the overall findings nor the data [9],[10]. Since publication, the data's reliability and heterogeneity have been called into question: nearly half of the observations are missing for low-income countries [11], making a reliance on modeled estimates and imputation essential. As Lu and colleagues acknowledge, there is only a 65% correlation between the two main data sources, WHO and IMF. In 29 country-year observations, the ratio between WHO and IMF estimates is greater than 10 (Table 1). In addition to questionable data, Lu and colleagues leave out of the analysis 51 countries that IHME previously analyzed as recipients of DAH, including Russia and much of Eastern Europe, Iraq, Afghanistan, the occupied Palestinian territory, Somalia, and several small Island states (Box 1) [12].

**Table 1:** Observations where the ratio of WHO to IMF estimates of government health expenditure from domestic sources as a percentage of GDP (GHE-S/GDP) is greater than 10.

Country	Ratio of WHO to IMF GHE-S
Central African Republic, 2002	1,600.98
Suriname, 2001, 2004, 1996, 2005, 2003, 1999	108.98, 104.12, 84.15, 35.08, 32.21, 15.52
Laos, 1998	54.20
Rwanda, 1996, 1995	44.57, 15.83
Cambodia, 2006, 2000	37.55, 23.27
Guinea, 2003, 2000	34.75
Burundi, 2002	33.84
Mozambique, 2004	24.78
Costa Rica, 1995, 1997, 2006, 2003, 2004, 2002, 1999	19.56, 18.16, 17.80, 16.47, 16.10, 15.94, 13.05
Malawi, 2000, 2003	13.43, 10.15
Niger, 1996	12.81
Laos, 1997	12.41
Fiji, 1998	11.58
Equatorial Guinea, 2000	10.93

WHO estimates exceed IMF estimates in about two-thirds of observations. However, there are also notable country-years in which WHO estimates are more than 10-fold lower than IMF estimates, including: Guinea-Bissau, 1995 (ratio of 0); Eritrea in 2003 (ratio of 0.047).

**Box 1. DAH-Receiving Countries Omitted from Study by Lu and Colleagues [6]**

Afghanistan

Albania

Belarus

Bosnia and Herzegovina

Bulgaria

Cook Islands

Croatia

Cuba

Dominica

Estonia

Falkland Islands

Gibraltar

Grenada

Honduras

Iraq

Kiribati

Korea, Democratic People's Republic

Latvia

Lithuania

Macedonia

Marshall Islands

Mayotte

Micronesia

Moldova

Montenegro

Montserrat

Myanmar

Nauru

Niue

Northern Mariana Islands

Palau

Palestinian Territory, occupied

Poland

Romania

Russian Federation

Saint Helena

Saint Kitts and Nevis

Saint Lucia

Saint Vincent and the Grenadines

Sao Tome and Principe

Serbia

Seychelles

Somalia

Timor-Leste

Tokelau

Tonga

Turks and Caicos Islands

Tuvala

Ukraine

Wallis and Fortuna

Yugoslavia

Even if we accept the concerns about data consistency and accept the highly imputed data, the relationship between DAH and GHE-S is not stable to the exclusion of a few data points. We replicated the author's fixed effects model (Arellano-Bover/Blundell Bond model). We confirmed their main results, but we further explored the sensitivity of the results to the exclusion of questionable data. The associations failed significance testing at *p* = 0.05 when excluding the lowest 10% of GHE-S using the IMF data and the lowest 20% of the WHO data.

Given the concerns about Lu and colleagues' model choice, we repeated the analysis using an alternative statistical model to assess the robustness of the relationship between DAH and GHE-S. We used ordinary least squares regression with country fixed effects, clustered by country, for the main model estimation of the association between DAH and GHE-S. We avoided random effects estimation because the aid literature suggests that the differences in the manner in which countries handle aid funds are structural (“fixed”) and idiosyncratic, so an exchangeability assumption seemed inappropriate. Countries have different means of interacting with donors: some require donors to buy into and contribute toward a national plan (e.g., India), while others allow donors freedom to implement projects with few constraints (e.g., Tanzania) [13]. Countries also have differences in national institutions that collect, disseminate, and report on foreign assistance. These fixed differences may be beneath the wide variation seen in country trends (Figure 2). Furthermore, donors take widely varying strategies toward liaising with government. For example, while World Bank funding largely goes through official government channels, the United States Government's President's Emergency Plan for AIDS Relief (PEPFAR) had largely bypassed recipient country budget-planning procedures in its effort to achieve a rapid scale-up of HIV/AIDS programs [14].

**Figure 2:** Widely divergent trends in the relationship between DAH and GHE-S in select countries. Both DAH and GHE-S are presented here as a percentage of GDP, with GHE-S based on IMF data. In Rwanda, GHE-S is effectively zero, regardless of DAH. In Lesotho, GHE-S appears to rise with DAH (aid is associated with additional GHE-S). Eritrea exhibits erratic response, while Zambia generally follows the predictions of Lu and colleagues about decreasing government expenditure with increasing DAH. Data source: IHME [2].

We tested the sensitivity of the results to the exclusion of observations from years where recipient governments were calculated to spend less than 0.01% of GDP from domestic sources on health. In a country with a GDP per capita of US$1,000, this means that the government is spending less than US$0.10 of non-donor money on health per capita. The IHME data show that GHE-S is less than 0.01% of GDP in 47 (out of over 1,200) country-year observations using IMF data and in 8 country-year observations using WHO data (Table 2). The linear association between DAH and GHE-S as percentage of GDP is not significant after excluding these observations. According to IMF data, Rwanda has had such near-complete displacement every year from 1997 to 2006. Cambodia, Ethiopia, and Guinea-Bissau follow a very similar trend to Rwanda, all showing near-complete displacement every year. If real, such complete displacement suggests alternative national priorities, and donors could seek alternative approaches to aligning their priorities with those of the recipient government. If we exclude these observations where GHE-S is less than 0.01%, there is no longer a statistically significant linear relationship between GHE-S and DAH.

**Table 2:** Country-years in which GHE-S/GDP <0.0001 in IMF and WHO data.

Country	Years Using IMF Data	Years Using WHO Data
Burundi	2002–2006	2003–2006
Cambodia	1995, 1998, 2003–2005	—
Central African Republic	2002, 2004	—
Comoros	2005	—
Ethiopia	2003, 2005, 2006	—
Guinea	2004–2006	—
Guinea-Bissau	2001–2004, 2006	1995, 2001, 2006
Laos	1999, 2005	2005
Madagascar	2004	—
Malawi	2004	—
Mozambique	1995–1997	—
Rwanda	1997–2006	—
Suriname	1995	—
Tanzania	2004–2006	—
The Gambia	2005	—
Zambia	2003–2004	—

If these data points are excluded, the relationship between GHE-S and DAH is no longer statistically significant.

Furthermore, linear regressions examining the association between DAH and GHE-S as a percentage of GDP when DAH to government is greater than or equal to 0.5% of national GDP are not significant. That is, countries that receive a substantial amount of DAH show little evidence of displacement. Notably, just under half of DAH is given to countries receiving greater than or equal to 0.5% of GDP as DAH (Table 3). DAH to governments is not displaced when aid makes a large (greater than or equal to 0.5% of GDP) contribution to health spending. This calls into question the argument that governments displace aid because they are not able to absorb it. It appears that aid displacement trends, even if we accept all the flawed data, are driven by those countries that receive very small amounts of aid for health, as the relationship is absent if we look at country-years in which aid makes up 0.5% of GDP or greater (Table 4).

**Table 3:** Country-years in which DAH equals or exceeds 0.5% of GDP.

Country	Years
Angola	1995, 2001
Armenia	2000
Benin	1999–2001, 2003, 2004
Bhutan	1997–2000
Bolivia	2003–2004
Burkina Faso	2000, 2001, 2005
Burundi	2002–2006
Cambodia	1995–1998, 2000–2006
Cape Verde	2001, 2003, 2005, 2006
Central African Republic	1999–2002, 2004
Chad	1997–2004
Comoros	1995–2000, 2002
Congo, Democratic Republic	2000, 2001, 2003–2006
Djibouti	1997–2000, 2005, 2006
Equatorial Guinea	2003–2004
Eritrea	1995–2006
Ethiopia	2001–2006
Fiji	2003
Ghana	2000–2006
Guinea	2006
Guinea-Bissau	1996–1998, 2000–2006
Guyana	2003–2006
Haiti	1995–2004
Kenya	2001–2006
Kyrgyzstan	2000, 2003–2006
Lao People's Democratic Republic	1999–2000, 2003–2006
Lesotho	2001–2006
Madagascar	2004–2005
Malawi	1995–2006
Mali	1995–2006
Mongolia	1999, 2001
Mozambique	1995–2006
Namibia	2002, 2006
Nepal	1998–2004
Nicaragua	1997–2006
Niger	1995–1997, 2004–2006
Papua New Guinea	1996, 2000–1005
Rwanda	1999–2006
Samoa	1998, 2001–2005
Senegal	1999–2005
Sierra Leone	2003–2006
Suriname	1995–1999, 2000–2005
Swaziland	2003, 2005
Tajikistan	2003–2004
Tanzania	1995–2006
The Gambia	2005, 2006
Trinidad and Tobago	2006
Uganda	1996, 1998–2006
Zambia	1996–2006
Zimbabwe	2003–2006

Limiting the analysis to these country-years (comprising 47% of all DAH) reveals no significant relationship between DAH and GHE-S.

**Table 4:** Summary of regressions, with GHE-S/GDP as dependent variable, DAH to governments/GDP as independent variable.

Models	IMF GHE-S Data		WHO GHE-S Data	
	Coefficient (SE)	*p*-Value	Coefficient (SE)	*p*-Value
**All observations**				
Arellano-Bover/Blundell Bond model	−0.40 (0.07)	0	−0. 45 (0.04)	0
Linear, country clustered	−0.39 (0.11)	0.001	−0.20 (0.19)	0.15
**Exclude if WHO to IMF GHE-S estimate >10 (flawed data)**				
Arellano-Bover/Blundell Bond model	−0.40 (0.07)	0	−0.46 (0.05)	0
Linear, country clustered	−0.17 (0.14)	0.232	−0.20 (0.18)	0.27
**Exclude if GHE-S <0.0001 (outlier and improbable data)**				
Arellano-Bover/Blundell Bond model	−0.32 (0.03)	0	−0.39 (0.03)	0
Linear, country clustered	−0.23 (0.14)	0.103	−0.20 (0.20)	(0.34)
**Exclude if DAH to government <0.5% of GDP (policy relevant)**				
Arellano-Bover/Blundell Bond model	−0.22 (0.10)	0.835	−0.25 (0.07)	0.001
Linear, country clustered	−0.23 (0.13)	0.103	−0.01 (0.25)	0.966

Note that linear regressions fail with modest exclusions.

SE, standard error.

## The Current Evidence on Aid Displacement Cannot Guide Policy

First, even if displacement does exist, there is no evidence that it is a bad thing. A large-scale empirical analysis found no evidence that non-fungible sectoral aid (that is, aid earmarked or otherwise dedicated to its intended purposes) works better than fungible aid, when “better” is understood as economic growth, spending in pro-poor sectors, or reductions in infant mortality [15]. In Vietnam's health sector, Wagstaff found that project-level outcomes are not harmed by displacement of government funding, suggesting that governments aim to shift spending to support projects where additional investments provide the greatest improvements [16]. Furthermore, as a recent analysis of health financing in Honduras, Rwanda, and Thailand showed that these countries increased their domestic spending from domestic sources in response to increases in donor funding, a finding based on close examination of country-spending that is at sharp odds with the cross-country conclusions [17]. This study also found that donors were likely to shift funds in the face of increasing resources from the Global Fund. This finding raises the possibility that some of the measured “displacement” is exogenous; that is, countries are shifting resources in response to anticipated, promised, or real changes in DAH. Aid displacement may be a reasonable approach for governments to improve the societal benefits of resource allocation decisions when development assistance is volatile or threatened. Even if we accept Lu and colleagues finding that DAH to NGOs undergoes less displacement (and thus, increases government health expenditure), this likely reflects the fact that NGOs are less likely to be burdened by the risks of aid volatility; and, since NGO salaries tend to be higher, they may drive up public sector health wages and in turn government expenditures (see Text S1 for an analysis of the vulnerability of this finding).

Given the concerns raised over data plausibility and completeness, conclusions about the mean relationship between DAH and government health spending should be called into question. While there does appear to be an association, it is too tenuous, too dependent on problematic model selection, and inconsistent (even among individual countries) to be used for policy or resource-allocation decisions. We show that there is no significant aid displacement when government health expenditures from domestic sources exceed 0.01% of GDP, and no evidence of aid displacement when DAH exceeds 0.5% of GDP (Table 4).

No statistical model can adequately compensate for systematically wrong and missing data. While Lu and colleagues have gathered the best available data, and have been fully transparent in sharing their datasets and methods, the reality is that we still lack a sufficient accounting of public financing on health to make any conclusions on overall trends. Of course, some displacement of aid from the health sector may occur. It would be rational for governments seeking to improve the distribution of limited national resources, and seeking to avoid interruptions in health service provision with annual fluctuations in aid to avoid a rapid rise in health sector spending. However, our findings should relieve donors of the need to make unrealistic demands on recipient governments, and of the pressure to divert resources to NGOs. While in some settings aid likely is displaced from the health sector, we call into question the assertions that donor health funds are being systematically displaced and misused.

## Supporting Information

Text S1 **Statistical supplement: aid displacement.**
(DOC)

## Abbreviations

DAH: in development assistance for health
GDP: gross domestic product
GHE: health expenditure
IHME: Institute for Health Metrics and Evaluation
IMF: International Monetary Fund
WHO: World Health Organization
